RETRACTED

# *Bacillus tequilensis* strain ‘UPMRB9’ improves biochemical attributes and nutrient accumulation in different rice varieties under salinity stress

**DOI:** 10.1371/journal.pone.0260869

**Published:** 2021-12-13

**Authors:** Rakiba Shultana, Ali Tan Kee Zuan, Mohd Rafii Yusop, Halimi Mohd Saud, Ahmed M. El-Shehawi

**Affiliations:** 1 Agronomy Division, Bangladesh Rice Research Institute, Gazipur, Bangladesh; 2 Department of Land Management, Faculty of Agriculture, Universiti Putra Malaysia, UPM Serdang, Selangor, Malaysia; 3 Institute of Tropical Agriculture and Food Security, Universiti Putra Malaysia, UPM Serdang, Selangor, Malaysia; 4 Department of Agriculture Technology, Faculty of Agriculture, Universiti Putra Malaysia, UPM Serdang, Selangor, Malaysia; 5 Department of Biotechnology, College of Science, Taif University, Taif, Saudi Arabia; Ghazi University, PAKISTAN

## Abstract

Soil salinity exert negative impacts on agricultural production and regarded as a crucial issue in global wetland rice production (*Oryza sativa* L.). Indigenous salt-tolerant plant growth-promoting rhizobacteria (*Bacillus sp*.) could be used for improving rice productivity under salinity stress. This study screened potential salt-tolerant plant growth-promoting rhizobacteria (PGPR) collected from coastal salt-affected rice cultivation areas under laboratory and glasshouse conditions. Furthermore, the impacts of these PGPRs were tested on biochemical attributes and nutrient contents in various rice varieties under salt stress. The two most promising PGPR strains, i.e., ‘UPMRB9’ (*Bacillus tequilensis* 10b) and ‘UPMRE6’ (*Bacillus aryabhattai* B8W22) were selected for glasshouse trial. Results indicated that ‘UPMRB9’ improved osmoprotectant properties, i.e., proline and total soluble sugar (TSS), antioxidant enzymes like superoxide dismutase (SOD), peroxidase (POD) and catalase (CAT). Moreover, ‘UPMRB9’ inoculated rice plants accumulated higher amount of nitrogen and calcium in tissues. Therefore, the indigenous salt-tolerant PGPR strain ‘UPMRB9’ could be used as a potential bio-augmentor for improving biochemical attributes and nutrient uptake in rice plants under salinity stress. This study could serve as a preliminary basis for future large-scale trials under glasshouse and field conditions.

## Introduction

Agriculture plays a pivotal role in human survival by fulfilling food demands of rapidly growing population of the world [1]. Moreover, it provides raw materials for numerous industries and directly or indirectly serves as a source of employment. However, current agricultural production is way lesser than the estimated food required for increasing global population [2]. Global climate changes are further causing decrease in agricultural production. Twenty two percent (22%) of the total cultivated areas of the globe and 33% of the total irrigated areas are affected by soil salinity, which is continuously increasing at an alarming 10% annual rate [3].

RETRACTED

Approximately 13% of the total landmass in Malaysia is occupied by coastal areas. The coastal areas span over 4.43 million ha out of which 57% is utilized for agriculture [4]. However, salinity is the major constraint in in coastal areas due to seawater intrusion [5]. Rice is third most important crop in Malaysia; however, its production is lower than consumption resulting in rice import. Rice self-sufficiency is ~75% with an average yield of 4.5 t ha^-1^ season^-1^. Rice production in Malaysia must be increased by 7 t ha^-1^ season^-1^ to fulfil the rice requirements of the country [6, 7]. Nonetheless, ~0.1 million ha of rice production areas in the country would be affected by salinity till 2056 [8]. Hence, appropriate management strategies are needed to mitigate the adverse impacts of salinity on growth and productivity of rice crop.

Plant growth promoting rhizobacteria (PGPR) can ameliorate the negative impacts of salinity on crop growth. The PGPRs improve physiological, biochemical, and metabolic of plants by increasing the accumulation/production of osmolytes, antioxidant enzymes and ion concentration [9, 10]. The PRGPRs have been exploited recently in numerous studies to improve plant growth of various species under stressful environments. The inoculation of *Bacillus drentensis* rhizobacteria strain significantly improved stomatal conductance, transpiration rate, and total chlorophyll content of mungbean [11]. In another study, inoculation of *Pseudomonas sp*. and *Bacillus lentus* mitigated adverse effects of salinity stress on basil plants through upregulation of antioxidant system, photosynthesis, and mineral contents [12].

Malondialdehyde (MDA) content rises in plants under salinity stress, which is originated from the oxidation of unsaturated fatty acids regulated by reactive oxygen species (ROS) [13]. Higher production of ROS initiates damage to membrane integrity due to unsaturated lipid components’ peroxidation, leading to membrane leakage and desiccation. Inoculation of PGPRs reduce malondialdehyde accumulation in plants under salinity stress [14]. Proline and total soluble sugar (TSS) contents are sensitive physiological indices acting as osmolytes to resist plant growth against oxidative damage. Salt-stressed plants could be protected through the regulation of proline, which acts as a scavenger for free radicals and buffering cellular redox potential. Improved TSS content in plants is another defense mechanism against salt stress. It has been reported that PGPRs significantly increase proline and TSS in wheat plants [15]. Moreover, the role of antioxidant system in protecting plants at a high level of salinity is crucial. Inoculation of PGPRs triggers the production of antioxidant enzymes, i.e., superoxide dismutase (SOD), peroxidase (POD), or catalase (CAT) to reduce the detrimental effect of ROS under salinity stress. The SOD acts as a potent scavenger of superoxide which forms hydrogen peroxide by destroying superoxide [16].

RETRACTED

Inoculation of salt resistant PGPRs could alleviate the adverse effects of salinity stress in rice plants. Therefore, it was hypothesized that inoculation of salt tolerant POGPR would reduce the adverse effects of salt stress on rice plants. In-depth analyses were conducted to determine the impacts of selected indigenous salt tolerant PGPR isolates on the regulation of biochemical metabolites under salt stress conditions in rice plants. The results would help to improve rice productivity in saline areas.

## Materials and methods

### Screening for salt-tolerance and plant growth-promoting properties of selected bacterial isolates

A total forty-four (44) bacterial strains were isolated from salt-affected coastal rice-cultivated areas in northern Malaysia (5^0^41’20.2"N 100^0^25’44.9"E and Jilid85^0^ 42’48.7"N 100^0^21’54.4"E). No permits were required to collect the samples as there were no endangered species involved in the study. Five of these 44 strains were selected based on their profuse growth on 1M of NaCl amended tryptic soy agar (TSA) (Sigma-Aldrich) media. These five bacterial strains were further tested for salinity tolerance and plant growth-promoting traits following the protocol of Shultana et al. [17] and Tan et al. [18]. The exopolysaccharide (EPS) of five bacterial isolates, i.e., ‘UPMRA4’, ‘UPMRB9’, ‘UPMRE3’, ‘UPMRE6’, and ‘UPMRG1’ were extracted following ethanol precipitation technique. The precipitated EPS was harvested and oven dried. Selected bacterial strains were tested for floc yield production by filtering the bacterial cultures grown in NaCl-amended TSB medium. Oven-dried filter paper was weighed, and floc yield was calculated. The selected bacterial strains were checked for biofilm formation following the microtitre plate-based protocol. Sodium uptake of selected isolates was determined following acid digestion. The estimation of bacterial sodium uptake was measured using Atomic Absorption Spectrophotometer (AAS) (Perkin Elmer, Analyst 400 AAS). The indole-3-acetic acid (IAA) production was measured by spectrophotometric method using salkowsky reagent as an indicator for color development. The colorimetric method was used for the phosphate solubilization assay in which Barton’s reagent was used as an indicator. The amount of available potassium solubilized by the selected strains was measured with AAS. The salt-tolerant nitrogen-fixing isolates were screened out by observing the halo zone diameter at different levels of NaCl. The promising bacterial isolates qualified for attaining the desired traits were identified previously using the partial sequencing of the 16S rRNA gene following the standard molecular identification method [19]. The identified strains ‘UPMRB9’ and ‘UPMRE6’ revealed their identity as *Bacillus tequilensis* (NCBI accession number: NR 104919.1) and *Bacillus aryabhattai* (NCBI accession number: NR 115953.1), respectively.

RETRACTED

### Soil preparation and fertilizer application

Soils were collected from Sawah Sempadan, Block D, Tanjong Karang, Selangor, Malaysia. The soil is classified as Bernam series with a pH of 4.23. The initial content of available nutrients was 0.62% N, 0.08% P, 0.29% K, 0.23% Ca, and 0.33% Mg. The soil was air-dried for two weeks and sieved through a 2 mm sieve. Afterwards, 20 kg soil was weighed, sterilized, and transferred to a non-drained plastic pail (30 cm diameter × 46 cm height). Chemical fertilizers namely urea, triple superphosphate (TSP), and muriate of potash (MOP) were applied at the rate of 170, 80 and 150 NPK kg ha^-1^, respectively based on the recommendations by the Department of Agriculture, Kuala Selangor, Selangor, Malaysia. The TSP and MOP fertilizers were applied as basal dosages, while urea was applied in 3 splits at 15, 45, and 60 days after transplanting (DAT).

### Seed surface sterilization and germination

Rice seeds were surface-sterilized following Miché and Balandreau [20] with slight modifications. The seeds were soaked in ethanol (95%) for 10 s, then ethanol was discarded, and seeds were soaked in 3% NaOCl for 1 min (Chlorox) following six washings with sterilized water. A glass Petri dish covered with moistened filter papers (3 layers) was used to germinate 20 surface-sterilized seeds. Sterile distilled water was added regularly to keep the filter paper (Whatman No 1) moist, and the germination percentage was recorded daily for 5 days, before transplanting.

### Preparation of bacterial inocula and in vitro application to rice plants

The selected PGPR strains were inoculated to three rice varieties, i.e., ‘BRRI dhan67’, ‘Putra-1’, and ‘MR297’, which has been identified as tolerant, moderately tolerant, respectively under 8 dSm^-1^ salinity [21]. A fully-grown bacterial culture was inoculated to Tryptic Soy Broth medium and shaken for 24 hours. The bacterial suspension (approximately 10^8^−10^9^ CFU mL^-1^) or sterile distilled water (as control) were inoculated onto 5 days-old rice seedlings and left to settle for 1h. One seedling of each variety was transplanted to plastic pails. Rice plants were re-inoculated at 14 days after transplanting (DAT) and sterilized distilled water was added as uninoculated control. The soil salinity level was adjusted to 8 dSm^-1^ using sodium chloride (NaCl) and the EC level was maintained throughout the experimental period.

RETRACTED

### Collection and preparation of leaf sample for biochemical analysis

Three randomly selected mature leaves from each plant were plucked and kept inside sealed plastic bags. The leaves were grounded immediately using liquid nitrogen and preserved in sealed plastic bags and stored in a freezer (-80°C).

Malondialdehyde (MDA) content was determined following the protocol of Stewart and Bewley [22] with slight modifications. The leaf’s proline content was measured following the method by Bates et al. [23]. Total soluble sugar was determined according to Yemm and Willis [24]. Superoxide dismutase (SOD) activity was determined by adopting according to Gupta et al. [25]. The POD activity was determined using a substrate known as guaiacol following Rao et al. [26]. Catalase (CAT) activity was studied according to Aebi [27].

### Plant tissue analysis

Plant tissue samples (above-ground plant parts) were over-dried at 70°C for 72h. Plant samples were ground using a plant grinder and the nutrient concentrations were determined using the standard nutrient analyses protocol [28]. The dried plant sample (0.25g) was taken into a 100 ml digestion tube and 5ml of H_2_SO_4_ (concentrated) was added to each digestion tube. All tubes were transferred to digestion block and digestion was allowed for 3 h at 360°C. The digestion process was inhibited for 30 min and to promote organic matter oxidation, and a few drops of 30% H_2_O_2_ were decanted to each digestion tube. The heating period was extended for another hour at 350°C. The clear and cooled digested samples were diluted to 100 ml and filtered using filter paper (Whatman no.42) and stored in plastic vials before analysis. The samples were used to determine N, P, K, Ca and Mg concentrations using Atomic Absorbance Spectrophotometer (AAS) (Perkin-Elmer, 400). The uptake of N, P, K, Ca and Mg was determined by multiplying the value with plant dry weight [29].

### Experimental design and statistical analysis

The experiment was laid out following factorial RCBD with five replications. Rice varieties were the main factor, while PFPR strains were regarded as sub-factor. The collected data on plant traits were tested for normality and data were found normally distributed. Therefore, 2-way Analysis of Variance (ANOVA) was used to test the significance among applied treatments. Means were compared by Tukey’s studentized range (HSD) test 5% probability where ANOVA indicated significant differences. The analyses were done on SAS 9.4 software.

RETRACTED

## Results

### Salt-tolerance and plant growth-promoting properties of bacterial isolates

Out of five tested strains, ‘UPMRB9’ produced the highest amount of exopolysaccharide (EPS) (22.81 g L^-1^) under 1M NaCl concentration (Table 1 and Fig 1). This strain also produced significantly higher biofilm (OD 1.36) and uptake a higher amount of sodium (21.58 mgL^-1^) than the rest of the strains. Meanwhile, ‘UPMRE6’ recorded the highest floc yield production (21.96 g L^-1^). The plant growth-promoting characters showed that isolate ‘UPMRB9’ produced significantly higher IAA (12.86 μg mL^-1^) than other strains and ‘UPMRE6’ accumulated the highest phosphate (27.73 μg mL^-1^) and potassium (6.93 mg L^-1^).

**Fig 1:** Exopolysaccharide driven aggregation of (a) ‘UPMRB9’ and (b) ‘UPMRE6’ under 1M NaCl concentration.

**Table 1:** Salt-tolerance and plant growth-promoting traits of selected bacterial isolates under 1M NaCl concentration.

Bacterial isolates	Salt-tolerance characters				Plant growth-promoting characters			
	EPS (g L^-1^)	Floc yield (g L^-1^)	Biofilm (590_nm_)	Sodium uptake (mg L^-1^)	IAA (μg mL^-1^)	P Solubilization (μg mL^-1^)	K Solubilization (mg L^-1^)	Nitrogen fixation
UPMRA4	13.32c	16.79b	0.62d	8.4c	10.08b	13.42b	3.22c	-
UPMRB9	22.81a	21.36a	1.36a	21.58a	12.86a	18.54b	4.75b	++
UPMRE3	15.54bc	8.80c	0.43e	2.4d	6.43c	12.69b	3.98bc	+
UPMRE6	20.88ab	21.97a	1.26b	13.86b	9.21b	27.73a	6.93a	++
UPMRG1	17.19abc	11.10c	1.13c	11.62b	10.97a	14.67b	3.98bc	++
MSD_(0.05)_	5.71	2.88	0.07	4.09	1.85	5.85	0.945	

Note: ’+’ indicates positive, ’-’ indicates negative; means having the same letter in a column do not differ significantly using tukey (HSD) at P>0.05.

### The impact of PGPR inoculation on biochemical attributes of rice varieties under salt stress

Bacterial inoculations significantly reduced the rice varieties’ malondialdehyde (MDA) contents under salt stress conditions. Inoculation of UPMRE6 to rice variety BRRI dhan67 and Putra-1 (5.72 nmol g^-1^ FW) significantly reduced the malondialdehyde content by 25.70% and 39.81%, respectively, while UPMRB9 significantly reduced the MDA content of MR297 variety by 25.37% (Fig 2).

**Fig 2:** Effect of bacteria inoculation on malondialdehyde content of rice varieties under salt stress. Means having the same letter within each variety do not differ significantly at the probability level 0.05 by Tukey (HSD).

RETRACTED

Bacterial inoculations significantly increased osmoprotectants [proline and total soluble sugar (TSS)] in all varieties under salt stress. Inoculation of ‘UPMRB9’ significantly increased proline content in variety ‘BRRI dhan67’ and ‘Putra-1’ by 140.17% and 144.86%, respectively, while ‘UPMRE6’ increased proline content of variety ‘MR297’ by 45.17%. The TSS in ‘BRRI dhan67’ and ‘MR297’ were increased by 93.27% and 77.72%, respectively with the inoculation of ‘UPMRE6’ and similar trends were observed for ‘UPMRB9’ inoculation in ‘Putra-1’ variety (Fig 3).

**Fig 3:** Effect of bacterial inoculation on proline (left) total soluble sugar contents (right) of rice varieties under salt stress. Means having the same letter within each variety do not differ significantly at the probability level 0.05 by Tukey (HSD).

Similar benefits were observed on the activities of antioxidant enzymes, i.e., SOD, POD and CAT for all varieties. Inoculation of bacterial isolate ‘UPMRB9’ resulted in higher SOD activity all varieties (Fig 4). The highest increment was noted for ‘Putra-1’ (89.70-unit mg^-1^ FW). Besides, inoculation of ‘UPMRE6’ significantly enhanced POD activity in ‘BRRI dhan67’ (54.22 μmol min^-1^ mg^-1^ FW) and ‘Putra-1’ (50.11 μmol min^-1^ mg^-1^ FW), whilst the highest amount of POD was noted for ‘MR297’ inoculated with ‘UPMRB9’ (Fig 5). Furthermore, variety ‘BRRI dhan67’ produced the highest CAT activity (18.41 μmol min^-1^ mg^-1^ FW) ‘UPMRB9’ inoculation. Similar trends were observed for ‘Putra-1’ and ‘MR297’ with an increment of 21.50% and 27.41%, respectively with ‘UPMRE6’ inoculation.

**Fig 4:** Effect of bacteria inoculation on superoxide dismutase (SOD) production in rice varieties under salt stress. Means having the same letter within each variety do not differ significantly at the probability level 0.05 by Tukey (HSD).

**Fig 5:** Effect of bacterial inoculation peroxidase (POD) and catalase (CAT) activity in rice varieties under salt. Means having the same letter within each variety do not differ significantly at the probability level 0.05 by Tukey (HSD).

Bacteria inoculations significantly increased nutrient uptake in all rice varieties. Inoculation with ‘UPMRB9’ to ‘BRRI dhan67’ and ‘MR297’ increased nitrogen (N) uptake by 39.88% and 158.46%, respectively. Similarly, ‘UPMRE6’ inoculation increased N uptake in ‘Putra-1’ variety by 83.72% (Table 2). Besides, phosphorus (P) uptake in ‘BRRI dhan67’ and ‘MR297’ was increased by 225.23% and 164.75%, respectively with ‘UPMRE6’ inoculation and ‘UPMRB9’ inoculation improved P uptake in ‘Putra-1’ by 81.96%. Furthermore, ‘UPMRB9’ significantly increased K uptake in ‘BRRI dhan67’ by 201.49%, while ‘UPMRE6’ increased K uptake in ‘Putra-1’ and ‘MR297’ by 276.47% and 123.87%, respectively. Similar trends were observed for Ca and Mg uptakes with 72.32–212.75% increase with inoculation of these strains.

RETRACTED

**Table 2:** Effect of bacteria inoculation on nutrient uptake in rice varieties under salt stress.

Variety	Nitrogen (N)			Phosphorous (P)			Potassium (K)			Calcium (Ca)			Magnesium (Mg)		
	(g plant^-1^)			(g plant^-1^)			(g plant^-1^)			(g plant^-1^)			(g plant^-1^)		
**Control**	**UPMRB9**	**UPMRE6**	**Control**	**UPMRB9**	**UPMRE6**	**Control**	**UPMRB9**	**UPMRE6**	**Control**	**UPMRB9**	**UPMRE6**	**Control**	**UPMRB9**	**UPMRE6**
**BRRI dhan67**	1.73b	2.42a	2.25a	1.07c	2.38b	3.48a	10.08c	30.39a	23.17b	1.7b	3.21a	2.53ab	1.33b	2.50a	2.38a
**Putra-1**	1.29c	1.87b	2.37a	2.55b	4.64a	3.45b	5.61c	13.93b	21.12a	1.77b	3.05a	2.77a	1.02c	1.84b	3.19a
**MR297**	1.30c	3.36a	1.94b	1.22c	2.72b	3.23a	4.86c	7.71b	10.88a	1.04b	2.04a	2a	1.14b	1.82a	2.21a

Means having the same letter within each variety do not differ significantly at the probability level 0.05 by Tukey (HSD).

## Discussion

Salt-tolerant PGPRs could play significant role augmenting plant growth under salt stress. Bacterial EPS and biofilm productions are two important salt-tolerance characteristics. The ‘UPMRB9’ produced high amount of EPS and significantly influenced bacterial biofilm formation. The EPS plays a critical role in forming biofilm which connects within bacterial cells. Higher availability of EPS-producing bacteria enhances nutrient and water uptake in rhizosphere; thus, establishes successful plant-microbe interactions [30]. The EPS can reduce negative effect of osmotic stress by increasing water content in plants; thus, augment fresh and dry weight of crop plants [31]. Bacterial cells within EPS layer are protected by biofilm which acts as a boundary between cells and surrounding saline environment. These associative properties cause the strain to absorb a high amount of sodium from the salt-amended medium, while maintaining a relatively high population. In this study, available Na^+^ in the soil was reduced by the EPS-producing bacteria which consequently alleviated adverse effects of salt stress in plants. This agrees with previous findings stating that ‘UPMRB9’ is a high producer of EPS and biofilm under 1.5M NaCl salinity [17]. This is also in line with Hong et al. [32] who demonstrated that the adhesive properties of EPS supported aggregate formation of bacteria with the soil particles and binds Na ions, thereby reducing sodium toxicity in plants. Sayyed et al. [33] stated that bacterial polysaccharides are acidic in nature and show high affinity towards certain ions. Kasim et al. [34] reported that higher concentrations of NaCl stimulated biofilm formation in *Bacillus spp*. where the highest peak was attained at 500 mM. These salt-tolerance characteristics of bacteria in the current study were supported by the SEM observation in a previous study, indicating that bacterial aggregation mediated by EPS production when exposed to saline conditions [19]. Genus *Bacillus* is abundantly present in the soil due to its ability to survive under several environmental stresses like UV radiation, desiccation, chemical damage, salinity etc. [35, 36]. The IAA production is an important plant growth-promoting trait in PGPR, as it is a signaling molecule in the regulation of plant development. In this study ‘UPMRB9’ produced high amount of IAA which posed beneficial effects to root growth and elongation, leading to better water and nutrients’ uptake. Bacterial cells could associate with plant root system to improve moisture-holding capacity and defense system against different abiotic stresses. The strain ‘UPMRE6’ showed better performance towards phosphorous and potassium solubilization. The PGPR can go through a range of processes to affect P transformation; thus, stimulates P availability as phosphate to plant roots [37]. Non-labile P reserve in the soil can be accessible to crops through the secretion of organic acids and hydrochloric ions regulated by phosphorus solubilizing bacteria (PSB). Several bacteria, including *Rhizobium*, *Pseudomonas*, *Enterobacter* and *Bacillus* are most effective P-solubilizers [38]. Moreover, some bacterial strains are well known to release K in its available form from K-bearing minerals in soils like *Acidothiobacillus sp*, *Bacillus edaphicus*, *Bacillus mucilaginosus*, *Ferrooxidans sp*, *Burkholderia sp* and *Paenibacillus sp*. [38, 39]. Besides, three bacterial strains, i.e., ‘UPMRB9’, ‘UPMRE6’, and ‘UPMRG1’ can fix atmospheric N under a high salinity. This agrees with Yan et al. [40] who showed that salt-tolerant PGPRs with N-fixing abilities could produce osmolytes to retain the turgidity and metabolism of cells in saline soils.

RETRACTED

Malondialdehyde (MDA) content is a good indicator of the extent of plant oxidative injury affected by salinity. Higher MDA content in cells increases the permeability of membrane and electrolytes outflows; thus, causes higher cell injuries. In the current study, rice variety ‘BRRI dhan67’ inoculated with ‘UPMRB9’ showed low electrolyte leakage under salt stress. This shows that cell membrane integrity can be protected by applying EPS-producing rhizobacteria that can act as barriers to prevent direct contact of sodium ion with plant roots and inhibit upward translocation of sodium ion. Cell membrane damage in various crops due to the generation of ROS and lipid peroxidation were shown in many previous studies [13, 14, 41–45].

Essential nutrients’ uptake in rice plant was influenced by bacterial inoculation. This has been reported in previous studies single or combined inoculation of *Lysinibacillus xylanilyticus* and *Bradyrhizobium japonicum* increased nutrient contents (P, K, Ca and Mg) in rice plants [7]. Crops inoculated with bacterial strains showed profuse vegetative growth with more surface area of roots for absorbing a higher amount of nutrients and water; thus, enhancing Ca and Mg uptake [46]. Earlier findings have indicated that PGPR colonizes plant roots and enhances root health by providing nutrients and in return, receives exudates from their associates [47]. These findings are in line with Dodd and Pe´rez-Alfocea [48] who illustrated that microbes could modify host plant physiology by producing a physical barrier around the roots and modifying the absorption of nutrients and toxic ions by roots (extensive rhizosheaths formation by bacterial exo-polysaccharides), or reduction of foliar noxious ions (Na^+^, Cl^-^) absorption; thus, improve the quantity of micro and macronutrients. It has been reported that multifarious halotolerant *K*. *variicola* SURYA6 acted as an effective bioinoculants for promoting plant growth by protecting plants from excess salt-induced damages, thus helped in accumulating higher soil nutrients in plants [49].

## Conclusion

The indigenous salt tolerant PGPRs, i.e., ‘UPMRB9’ and ‘UPMRE6’ improved biochemical attributes and nutrient uptake in rice under salinity stress. These are due to their multiple salt-tolerance and plant growth-promoting characteristics which are crucial in maintaining normal physiological functions and regulations of antioxidant system under salt stress. These bacterial strains could be a used as promising biofertilizer inoculum to improve growth and yield of rice in saline areas. However, extensive field trials are needed before making a general recommendation.
